RETRACTED

# Effects of Core Stabilization Training on the Cobb Angle and Pulmonary Function in Adolescent Patients with Idiopathic Scoliosis

**DOI:** 10.1155/2022/4263393

**Published:** 2022-07-31

**Authors:** Kexin Qi, Haidong Fu, Zhen Yang, Lingqi Bao, Yinxin Shao

**Affiliations:** ^1^Department of Physical Education and Research, Changchun University, Changchun 130000, China; ^2^Academic Affairs Office, Changchun University, Changchun 130000, China; ^3^Luoyang Institute of Science and Technology, LuoYang 471023, Henan, China; ^4^Graduate School of Changchun University, Changchun 130000, China

## Abstract

**Objective:**

To observe the effects of core stabilization training on the Cobb angle, respiratory muscle strength (maximum inspiratory pressure, MIP; maximal expiratory pressure, MEP), and pulmonary function (forced vital capacity, FVC; forced expiratory volume, FEV1.0; FEV1.0/FVC%) in adolescent patients with idiopathic scoliosis (AIS) and offer practical-based evidence for the rehabilitation treatment for AIS patients.

**Methods:**

36 AIS patients were assigned to the core stability training (CST) group (*n =* 18) and control group (*n* = 18); the CST group participated in three sessions of core stabilization exercise per week for 12 weeks and the control group did not perform regular physical training during 12 weeks of study. Then, the Cobb angle, respiratory muscle strength (MIP and MEP), and pulmonary function (FVC, FEV1.0, and FEV1.0/FVC%) were measured before and after core stabilization training.

**Results:**

After 12 weeks of core stabilization training, compared with the pretest, the Cobb angle showed a significant decrease, FVC, FEV1, MIP, and MEP a significant increase (*P* < 0.01 respectively), and there was no statistical difference in FEV1/FVC in the CST group; there was no significant difference (*P* > 0.05 respectively) before and after an experiment in the control group except MEP decreased significantly (*P* < 0.01, *P* < 0.05). After 12 weeks of core stabilization training, compared with the control group, the Cobb angle significantly decreased (*P* < 0.01), FVC, FEV1, MIP, and MEP significantly increased (*P* < 0.05 respectively) in the CST group, but there was no significant difference (*P* > 0.05, respectively) in FEV1/FVC between the control group and CST group.

**Conclusions:**

Core stabilization exercise can be considered to have a positive effect on the normal physiological curvature of the spine in AIS patients, as it decreases the Cobb angle and strengthens respiratory muscle strength and pulmonary function.

## 1. Introduction

Scoliosis is a kind of skeletal muscle disease with spinal deflection or rotation; it is a generic term for a group of different diseases of the spine, thoracic, and trunk shape and position caused by a change in composition, which often occurs in the period of sudden growth before puberty [1]. Based on the age of presentation, scoliosis is further categorized as infantile, juvenile, or adolescent idiopathic. Adolescent idiopathic scoliosis (AIS) accounts for the majority of the three categories, presents at age ten, and lasts till the end of growth, and approximately 80% of scoliosis patients are AIS [2]. In worldwide, the prevalence of AIS ranges from 0.93% to 12%, and the incidence and severity of spinal curvature in girls are higher than those in boys [3]. Studies have shown that scoliosis can lead to decreased spinal movement, weakness of muscles near the spine, and balance dysfunction [4]. In addition, nearly two-thirds of scoliosis patients (Cobb angle >40°) are usually accompanied by restrictive abnormal breathing patterns which cause external deformities and reduce respiratory muscle contraction, limit the movement of ribs and trunk, and result in pulmonary dysfunction and respiratory dysfunction [5]. Moreover, Kato et al. [6] believed that asymptomatic patients with mild scoliosis might not have any respiratory dysfunction at rest, but there were some reports of abnormal ventilation mode and decreased respiratory muscle strength in mild scoliosis, and pulmonary dysfunction could be gradually aggravated with further deformity of the spine. Therefore, to prevent further spinal deformity, early intervention is very important for AIS patients.

RETRACTED

The treatment methods of AIS include surgical treatment (Cobb angle ≥40°) and conservative treatment. The traditional exercise treatment methods for scoliosis include posture exercise, stretching exercise, and muscle strength enhancement training [7]. Research shows that exercise rehabilitation intervention should be carried out as soon as possible for AIS patients, and exercise therapy in AIS is considered to be an important method to maintain spinal function, which can effectively prevent the development of scoliosis [8]. Recent studies have found that compared with traditional training, core stability training has a better effect on reducing rotation deformity and pain in AIS patients, which suggests that core stability training is an effective method for early treatment of AIS [9]. It is also reported that chest flexion will weaken respiratory muscles and reduce cardiopulmonary function, and core stability training can help abdominal breathing and improve pulmonary function by increasing the contraction of the diaphragm and transverse abdominal muscle [10]. Therefore, it can be considered that core stability training may have a more positive impact on spinal column morphology and pulmonary function in AIS patients. Based on the above assumptions, the current study observed the effects of 12 weeks of core stability training on Cobb angle, respiratory muscle strength, and pulmonary function in AIS patients, to provide a theoretical basis for the intervention of core stability training in AIS patients.

RETRACTED

## 2. Object and Methods

### 2.1. Research Object

According to the questionnaire “Screening for scoliosis abnormalities in children and adolescents” in September 2020 a professional physician assessed the spinal morphology of middle school girls in Changchun City, Jilin Province. All subjects participated in the screening with informed consent. Finally, professional doctors took the whole spine X-ray as the basis for diagnosis. Specific inclusion criteria are as follows: Cobb angle is 10–30° and has never undergone regular exercise therapy, surgical correction, and wearing braces, without lung disease, congenital chest deformation or rib fracture, and contraindications to exercise/physical activity. According to the above criteria, a total of 38 female middle school students met the criteria, including 20 students with thoracolumbar double bending and 18 students with thoracolumbar bending. Then, 38 AIS female middle school students were randomly divided into core stabilization training (CST group; *n* = 20) and control group (*n* = 18, only receiving regular evaluation guidance). All participants signed informed consent before the trial (in addition, 2 participants in the CST group stopped the rehabilitation plan for personal reasons). There was no significant difference in age, height, and weight between the two groups before exercise intervention (*P* > 0.05). The basic information of the subjects is given in Table 1.

### 2.2. Research Methods

#### 2.2.1. Exercise Intervention Program

The core stability training program is designed based on previous studies [10]; all participants performed the core stability training for 12 weeks (3 sessions per week, 60 min each session). Each session includes 10 minutes of warm-up and 5 minutes of relaxation (both stretching and posture exercises of large muscle groups) and 45 minutes of core stability exercise intervention. All movements are carried out under the supervision of professional teachers to ensure that all movements are accurate.

Core stability exercises include unstable equipment exercises (such as balance pad and Swiss ball), back bridge exercise, side bridge exercise, prone two-point support, supine bending and supine leg lifting, trunk curling, and cat camel stretching exercises; each type of exercise was conducted in 3 sets of 12 repetitions. During exercise, the polar table monitors the exercise intensity at any time.

RETRACTED

#### 2.2.2. Cobb Angle Measurement

The digital diagnostic equipment of Philips was used to examine the whole spine X-ray plain film (posterior-anterior position and lateral position) of 36 subjects before and after exercise intervention. Posterior-anterior position: the patient stands naturally, his feet are shoulder width apart, his eyes look straight ahead, and his hands hang down naturally on both sides of his body. Lateral position: the patient stands naturally with elbow flexion and shoulder hugging, to avoid the overlap of upper limb and spine during shooting.

Cobb angle was measured by a radiologist alone. The Cobb angle of the thoracolumbar spine was measured by measuring the X-ray photos of the spine before and after the subject's standing position. Draw a straight line along the upper endplate of the cephalic end vertebra and the lower endplate of the caudal end vertebra, respectively, and then make the vertical line of the two lines. The intersection angle is the Cobb angle. The maximum Cobb angle is taken for patients with thoracolumbar double curvature.

#### 2.2.3. Pulmonary Function Measurement

Before and after exercise training, the pulmonary function of the subjects was measured with a portable pulmonary function tester (Anhui Institute of Electronic Science), which was evaluated by a rehabilitation expert. The specific methods are as follows: the basic information of the subjects (name, gender, and age) was input before the test. During the test, the subjects relaxed, sat up straight, clamped the nose clip, and wrapped the blowing mouth with their lips without air leakage. Pulmonary functions include forced vital capacity (FVC), forced expiratory volume (FEV1.0), and the percentage of forced expiratory volume in forced vital capacity in the first second (FEV1.0/FVC%).

Respiratory muscle strength was assessed by maximum inspiratory pressure (MIP) and maximum expiratory pressure (MEP), respectively. During the test, the patient takes the sitting position, closes the nasal cavity with the nasal clip, holds the blowing mouth, and puts the blowing mouth close to the lips to prevent air leakage. Using abdominal breathing, the patient exhaled the air in the lung as much as possible, took a deep breath quickly after exhaling, and recorded MIP (cm H_2_O); the patient exhales quickly and forcefully after the maximum deep inhalation and then recorded MEP (cm H_2_O), repeat for 3 times, and take the average value.

### 2.3. Statistical Analysis

All experimental data were presented as mean ± standard deviation. SPSS 21.0 statistical software was used for statistical analysis. The paired sample *t*-test was used for the data of the control group and CST group before and after the experiment. An independent sample *t*-test was used for the difference between the groups before and after the exercise (control group and CST group). The significance level (*α*) was set to *P* < 0.05.

RETRACTED

## 3. Results

### 3.1. Effect of Core Stability Training on Cobb Angle in Patients with AIS

Table 2 provides that after 12 weeks of core stability training intervention, the Cobb angle of AIS patients in the CST group decreased significantly compared with that before exercise (*t* = 14.981, *P* < 0.01), with a decreased range of 15.50%. The Cobb angle of AIS patients in the control group increased compared with that before the experiment, but there was no significant difference in the Cobb angle between the before and after the experiment (*t* = −0.524, *P* > 0.05). There was no significant difference in Cobb angle between the two groups before exercise (*P* > 0.05). After 12 weeks of core stability training intervention, the Cobb angle of AIS patients in the CST group decreased significantly compared with the control group (*t* = 6.479, *P* < 0.001).

### 3.2. Effect of Core Stability Training on Respiratory Muscle Strength in Patients with AIS

Table 3 provides that after 12 weeks of core stability training intervention, compared with before exercise, MIP and MEP in the CST group increased significantly (*T* values were −9.072 and −5.250, respectively, *P* < 0.01); compared with that before the experiment, MEP of AIS patients in the control group decreased significantly (*t* = 3.688, *P* < 0.01), but there was no significant change in MIP (*t* = 0.313, *P* > 0.05). After 12 weeks of core stability training intervention, compared with the control group, MIP and MEP of AIS patients in the CST group significantly increased (*t* = −4.261, *P* < 0.001, *t* = −3.762, *P* < 0.001).

### 3.3. Effect of Core Stability Training on Pulmonary Function in Patients with AIS

Table 4 provides that after 12 weeks of core stability training, FVC and FEV1 in the CST group increased significantly compared with those before training (*T* values were −11.335 and −7.580, respectively, *P* < 0.01), and there was no significant difference in FEV1/FVC before and after training (*t* = −1.632, *P* > 0.05). There was no significant difference in the above indexes in the control group before and after the experiment (*P* > 0.05).

There was no significant difference in lung function between the two groups before core stability training (*P* > 0.05). After core stability training, FVC and FEV1 in AIS patients in the CST group increased significantly compared with the control group (*t* = −2.767, *P*=0.009; *t* = −3.434, *P*=0.002), while there was no significant difference in FEV1/FVC between the control group and CST group after core stability training (*t* = −1.198, *P*=0.052).

RETRACTED

## 4. Discussion

### 4.1. Effect of Core Stability Training on Cobb Angle in Patients with AIS

Recent studies found that the importance of core stability training for the improvement of spinal morphology in patients with scoliosis has been confirmed because it can stabilize the spine in the cooperation between deep and surface muscles, and it is effective in controlling a person's movement to maintain the neutral position of the spine [9]. Akodu et al. [11] believe that core stability training can correct spinal dislocation by improving neuromuscular control and enhancing the strength and endurance of trunk and pelvic floor muscles which has an obvious rehabilitation effect on low back pain and dysfunction in patients with chronic low back pain. However, there are few studies on the rehabilitation effect of core stability training on scoliosis. Park et al. [12] conducted 10 weeks of core stability training on 51 scoliosis students and found that the core stability training significantly reduced the lumbar Cobb angle of scoliosis students. Noh et al. [13] found that exercise intervention for 3.5–4 months (60 min/session, 2-3 sessions a week), including stretching exercise and back muscle strengthening training can significantly reduce the Cobb angle of AIS patients which suggested that muscle strengthening training could curb the development of scoliosis and prevent the aggravation of symptoms. In addition, Wang [14] conducted medical gymnastics intervention on AIS patients (5 lumbar scoliosis and 5 thoracic scoliosis, respectively) for 3 months. The results showed that the effective rate of medical gymnastics (core strength training and posture correction) on the correction of single thoracolumbar AIS patients was 88% and that of single lumbar AIS patients was 92%, suggesting that orthopedic gymnastics has a good intervention and correction effect on AIS patients, and the effect is slightly better for single waist bending type than single chest bending type. Meta-analysis showed that early exercise rehabilitation interventions for AIS patients with Cobb (10°–25°) should be performed to achieve good results, while AIS patients with Cobb angle ranging 30°–50 and above 50° had only moderate results [15].

AIS patients selected in this study include double bending type and chest bending type, and the average value of Cobb angle is (23.81° ± 2.46°) and belongs to mild and moderate AIS patients. AIS patients are given 12 weeks of core stability training which mainly conducted strength and stability training for core muscles and their deep small muscles and the body is in an unstable state with the help of a Swiss ball and balance pad to enhance the input of proprioception, recruit more core muscles, and increase the muscle strength of the convex side. So, core stability training may improve the asymmetric stress and let the body form and continuously strengthen the memory of the correct posture, to slow down the development of scoliosis and repair the curvature of the spine by enhancing the muscle strength of the convex side and stretching the muscles, ligaments, and other soft tissues of the concave side under long-term tension. The results showed that after 12 weeks of core stability training, the Cobb angle of AIS patients in the CST group decreased significantly, and the Cobb angle of the CST group also decreased significantly when compared with the control group. In addition, the current study also found that during the 12-week experiment, the Cobb angle in the control group increased from (23.88° ± 2.37°) to (24.00° ± 2.45°), suggesting that AIS patients are at risk of aggravating spinal deformity without any treatment. However, exercise intervention time is very important. Some scholars suggested that exercise therapy for AIS patients should last for at least 6 months or more, which has a greater impact on the Cobb angle [6]. Therefore, future studies should extend the intervention time of core stability training and verify the duration of the rehabilitation effect of core stability training on AIS patients.

RETRACTED

### 4.2. Effect of Core Stability Training on Pulmonary Function in Patients with AIS

Impaired pulmonary function in AIS patients has been fully confirmed. The maintenance of normal respiratory function requires normal thoracic volume and the relaxation and contraction activities of the diaphragm and intercostal internal and external muscles. Scoliosis often causes deformities of the spine and thorax which result in compression of lung tissue, imbalance of intercostal muscles on both sides, a decline of respiratory muscle strength, and reduction of the chest wall and lung compliance, thus affecting lung ventilation function [16]. Lung function is generally determined by respiratory muscle strength, chest compliance, airway resistance, and elastic recoil of the lung. FVC (forced vital capacity refers to the maximum amount of air that can be exhaled as soon as possible after trying to inhale), FEV1.0 (expiratory volume in the first second of starting exhalation), FEV1/FVC% (an important index to judge pulmonary ventilation function, the normal value is 83%), MIP and MEP are commonly used to evaluate pulmonary function in patients with AIS [17]. Most scholars have found that FVC, FEV1, MIP, and MEP of AIS patients are significantly lower than those of healthy adolescents [18, 19]. Ran [20] obtained the same results; compared with normal subjects, patients with congenital and idiopathic scoliosis had FEV1.0 and FVC decreased significantly, showing restrictive ventilation dysfunction characterized by decreased lung volume. Fabian et al. [21] found that MIP, MEP, and FVC in patients with mild AIS (Cobb angle 10–20°) decreased significantly when compared with healthy adolescents, and FVC was significantly correlated with respiratory muscle strength, which suggested that patients with mild AIS had mild pulmonary dysfunction earlier and needed early intervention to prevent further deterioration and reduce its impact on adolescent health.

RETRACTED

The traditional exercise therapy for scoliosis includes posture exercises and muscle strengthening exercises. It is effective for patients with mild scoliosis or in combination with orthopedic and traction therapy. Amăricăi et al. [22] performed 12-week physical therapy (muscle stretching exercise and intensive exercise, breathing training, and core strength training) on mild and moderate AIS patients (Cobb angle of 10–35°), and the results showed that FVC, inspiratory ability, FEV1, expiratory reserve capacity, and 6-minute walking test of AIS patients significantly improved. Moreover, Mustafaoglu et al. [23] found that a 6-week core stability exercise can significantly improve the pulmonary function (FVC, FEV1, and maximum expiratory flow) and respiratory muscle strength (MIP and MEP) of drug abuse adolescents. In this study, AIS patients were given core stability training for 12 weeks. The results showed that FVC, FEV1, MIP, and MEP significantly increased in AIS patients after 12 weeks of core stability training compared with those before exercise, but the ratio of FEV1/FVC had no significant change. Compared with the control group, the VC, FEV1, MIP, and MEP of the CST group increased significantly after 12 weeks of core stability training, and there was no significant difference in FEV1/FVC between the CST group and the control group, indicating that core stability training can improve the pulmonary function of AIS patients to a certain extent. The research shows that core stability training can stabilize the deep muscles of the lumbar spine, abdominal muscles, lower back and middle back, and the hip muscles of the pelvis and control the intraabdominal pressure which plays an important role in breathing and stabilizing the trunk [24]. Therefore, the improvement of lung function in AIS patients by 12 weeks of core stability training may be related to the activation of core muscles (diaphragm and transverse abdominal muscle), the increase of intraabdominal pressure, and the reduction of intrathoracic pressure and the increase of ventilation by contracting the abdominal wall. Moreover, core stability training can stimulate the plasticity and symmetrical development of the trunk by stretching shortened muscles and enhancing trunk muscles, which enhance the muscle strength of respiratory muscles and muscles around the spine and improve the stability and symmetrical development of the trunk, to improve the pulmonary function of AIS patients. Most scholars believe that the severity of spinal deformity (the size of Cobb angle), the number of spinal affected segments, the position of the curve, and the loss of normal thoracic kyphosis are related to pulmonary function [25]. In previous studies, the relationship between spinal deformity and pulmonary function was reported. The study found that the degree of the thoracic curve (thoracic Cobb angle) was significantly negatively correlated with FVC and FEV1, and the patients with a large thoracic Cobb angle had a more obvious decline in FEV1 and FVC. Some scholars believe that the Cobb angle of patients is significantly negatively correlated with lung function. Generally, scoliosis within 40° (Cobb angle) has little impact on lung function, scoliosis >70° (Cobb angle) will cause severe restrictive ventilation dysfunction, and patients with >100° (Cobb angle) or large rotation angle will even have pulmonary insufficiency [26]. The average Cobb angle of AIS patients selected in this study was (23.81° ± 2.46°) degrees, including double bending type and chest bending type. The mean value of FEV1/FVC is (0.81 ± 0.06)%, which is close to the normal range (the normal value is 0.83), which is the same as the above results, indicating that scoliosis Cobb angle <40° has little effect on pulmonary function. Therefore, there was no significant change in FEV1/FVC in the experimental group after 12 weeks of core stability training, and there was no significant difference in FVC and FEV1/FVC between the experimental group and the control group, which may be related to the severity and type of scoliosis in AIS patients in this study.

RETRACTED

## 5. Summary

To sum up, 12-week core stability training has a positive impact on the physiological curvature of the spine of AIS patients, which can significantly reduce the Cobb angle of AIS patients and enhance the respiratory muscle strength and lung function of AIS patients. However, subsequent studies need to verify the duration of the rehabilitation effect of core stability training on AIS patients.

## Figures and Tables

**Table 1:** Physical characteristics of subjects ($\bar{x}\pm s$).

	*n*	Age (year)	Height (m)	Weight (kg)
Control group	20	13.61 ± 1.33	1.55 ± 0.03	47.68 ± 2.45
CST group	18	13.94 ± 1.30	1.56 ± 0.03	49.04 ± 1.91

**Table 2:** Results of Cobb angle pre and post core stabilization training in AIS ($\bar{x}\pm s$).

Group	*n*	Pretreatment	Posttreatment	*t* value	P value
Control group	18	23.88 ± 2.37	24.00 ± 2.45	−0.524	0.607
CST group	18	24.06 ± 3.84	20.33 ± 3.61^##ΔΔ^	14.981	<0.001

^##^ *P* < 0.01, comparison before and after the experiment; ^ΔΔ^*P* < 0.01, vs. the control group.

**Table 3:** Results of MIP and MEP pre and post core stabilization intervention in AIS ($\bar{x}\pm s$).

Respiratory muscle strength	Group	Pretreatment	Posttreatment	*t* value	*P* value
MIP (cm H_2_O)	Control group	61.12 ± 8.99	60.94 ± 7.77	0.313	0.758
	CST group	60.89 ± 8.03	74.11 ± 9.87^##ΔΔ^	−9.072	*<*0.001

MEP (cm H_2_O)	Control group	72.67 ± 6.90	71.33 ± 7.36^##^	3.688	0.002
	CST group	71.61 ± 8.51	84.61 ± 13.04^##ΔΔ^	−5.250	*<*0.001

^##^ *P* < 0.01, comparison before and after the experiment; ^ΔΔ^*P* < 0.01, vs. the control group.

**Table 4:** Results of pulmonary function pre and post core stabilization training in AIS ($\bar{x}\pm s$).

Pulmonary function	Group	Pretreatment	Posttreatment	*t* value	*P* value
FVC (ml)	Control group	2494.83 ± 269.13	2463.44 ± 291.62	0.266	0.783
	CST group	2478.33 ± 374.09	2756.50 ± 341.85^##ΔΔ^	−11.335	*<*0.001

FEV1 (ml)	Control group	2043.39 ± 205.19	2006.11 ± 266.59	0.381	0.708
	CST group	2026.94 ± 299.07	2322.33 ± 285.67^##ΔΔ^	−7.580	*<*0.001

FEV1/FVC	Control group	0.82 ± 0.03	0.81 ± 0.04	0.587	0.565
	CST group	0.82 ± 0.06	0.84 ± 0.04	−1.632	0.121

^##^ *P* < 0.01, comparison before and after the experiment; ^ΔΔ^*P* < 0.01, vs. the control group.

## Data Availability

The data used to support the findings of this study are available from the corresponding author upon request.
